# Necrosis Following Dermal Injection of Lyophilized Exosomes: A Case Report

**DOI:** 10.1111/jocd.70387

**Published:** 2025-08-18

**Authors:** Salma AlBargawi

**Affiliations:** ^1^ Department of Dermatology College of Medicine, Imam Mohammad Ibn Saud Islamic University Riyadh Saudi Arabia

**Keywords:** acne scars, dermal injection, exosome, necrosis

## Abstract

**Background:**

Exosomes are extracellular vesicles produced by virtually all cell types. In dermatology, exosomes have garnered significant attention for their potential applications in skin restoration and rejuvenation. Despite their widespread marketing in aesthetic medicine, no exosome product is currently approved for dermal injection, and their safety profile remains unclear.

**Aims:**

To report a rare case of ischemic necrosis following dermal injection of lyophilized exosomes for acne scar treatment and to emphasize the potential risks of unregulated aesthetic products.

**Patient/Methods:**

A 38‐year‐old male presented with painful ulcerated papules and dusky discoloration on both cheeks 3 days after receiving multiple intradermal injections of Korean‐manufactured exosomes. Clinical findings were consistent with ischemic necrosis. Laboratory tests including ANA, CBC, and LFTs were unremarkable. The patient declined biopsy. Supportive care and subsequent laser treatments were performed to manage the resulting atrophic scars and pigmentation.

**Results:**

At 2 weeks, eschars spontaneously sloughed off without secondary infection. However, the patient developed significant atrophic scarring with hyperpigmentation. Three laser sessions (CO_2_ followed by Er:YAG) yielded only modest improvement. The clinical progression and absence of systemic findings indicated localized vascular compromise, likely due to the exosome product.

**Conclusions:**

This case highlights a serious, underreported complication of unapproved exosome‐based injectable therapies. The ischemic necrosis and resulting scarring underscore the importance of regulatory oversight and clinical caution when using such products. Further research and safety evaluation are essential before exosomes can be routinely used in dermatologic practice.

## 1 Introduction

Acne scars are a common concern frequently encountered in dermatology practice. Among the various types of acne scars, atrophic scars are the most prevalent, resulting from insufficient collagen production during the wound healing process. Exosomes are extracellular vesicles, typically 30–150 nm in size, and are produced by virtually all cell types [1]. In dermatology, exosomes have garnered significant attention for their potential applications in skin restoration and rejuvenation through extracellular matrix production and matrix metalloproteinases (MMP) inhibition [2]. The most common source of exosomes used in aesthetic medicine is human mesenchymal stem cells (MSCs). Current marketed exosome products have shown promise in enhancing skin texture, reducing wrinkles, and improving overall skin health, largely attributed to their proposed anti‐inflammatory and regenerative properties [3]. However, no exosome product has received regulatory approval for injection or the treatment of any medical condition.

## 2 Case Description

A 38‐year‐old male presented with painful skin lesions on the cheeks 3 days after undergoing multiple dermal injections of exosomes at a different center. We obtained signed informed procedural consent prior to treatment and for the publication of this case report and accompanying images. After the patient followed up with the treating clinic, it was confirmed that the injections were performed by a non‐dermatologist physician using Korean‐manufactured exosomes (Curstem C20, Kangstem Biotech, South Korea) to improve the appearance of acne scars. The product label claims that it contains 200,000 ppm of human blood cord conditioned media as lyophilized powder, which is then reconstituted with normal saline. Clinical examination revealed multiple punched‐out, ulcerated papules on the cheeks, with slightly raised eschars and dusky purple discoloration (Figure 1). No significant swelling, pus, or discharge was observed. Laboratory tests, including antinuclear antibody (ANA), liver function test (LFT), and complete blood count (CBC), were within normal ranges. The patient's medical and dermatological history was unremarkable.

**FIGURE 1:** (A): Left cheek showing multiple punched‐out, ulcerated papules with raised eschars and dusky purple discoloration, 3 days after the dermal injection of exosomes. (B): Right cheek dusky purple discoloration.

At the 2‐week follow‐up, the eschars gradually sloughed off without signs of secondary infection, and the erythema subsided (Figure 2A). However, the scars healed in a noticeably atrophic manner with hyperpigmentation. The patient underwent a session of fractional carbon dioxide laser treatment, followed 6 weeks later by two sessions of erbium‐doped yttrium aluminum garnet (Er: YAG) laser, spaced 4 weeks apart. Modest improvement was observed in scar depth, pigmentation, and overall appearance (Figure 2B). Nevertheless, no complete resolution of the scars or pigmentation occurred.

**FIGURE 2:** (A): Two‐week follow‐up showing noticeable atrophic scarring and hyperpigmentation after the initial presentation. (**B**): Four weeks post CO2 fractional laser treatment, demonstrating some scar depth and texture improvement. (C): Ten weeks after two Er: YAG laser treatments, showing modest improvement from initial presentation, with ongoing atrophic scarring despite laser treatments.

The clinical presentation and progression were consistent with ischemic necrosis, likely due to vascular compromise. Histopathological testing could have confirmed the diagnosis; however, the patient declined further interventions. This case highlights a rare adverse effect of exosome‐based therapies and underscores the need for stringent regulatory compliance when using unapproved products.

## 3 Discussion

Exosomes have emerged as promising therapies in dermatology, particularly for their proposed regenerative and anti‐inflammatory properties. Despite their increasing use in aesthetic medicine, their safety profile remains largely unexplored. Currently, no exosome product is approved by regulatory bodies for dermal injection or the treatment of any condition. Although several countries appropriately restrict injecting unapproved products, this is not the case in some parts of Asia and the Middle East. Nevertheless, the manufacturer recommends never injecting their product but instead topically applying it and using a microneedling device.

This case presents a significant complication involving the intradermal injection of an exosome product, resulting in ischemic necrosis, which subsequently led to worsened scarring and hyperpigmentation. Clinically, the patient developed multiple punched‐out, ulcerated papules with raised eschars and dusky, purple discoloration 3 days after receiving dermal injections of exosomes. Infection was ruled out due to the absence of significant swelling, pus, or discharge. Additionally, normal laboratory findings, including ANA, LFT, and CBC, excluded systemic involvement or conditions such as autoimmune vasculitis or other inflammatory processes. The lack of systemic symptoms further supported a vascular compromise rather than a systemic reaction. These findings are consistent with tissue ischemia and necrosis.

Necrosis resulting from cosmetic injectables is a rare complication; however, it is most commonly associated with soft tissue fillers, which can cause vascular compromise [4]. Cases of HA‐based filler vascular compromise are typically managed with hyaluronidase and often resolve without long‐term sequelae. In this case, the necrosis may have resulted from localized vascular injury, pressure effects, or microembolization caused by the exosome product.

In the literature, only one similar case has been reported, involving a 36‐year‐old man who developed painful facial rashes on both cheeks after receiving multiple intradermal injections of a similar exosome formulation [5]. The lesions in that case exhibited notable resolution, ultimately leaving atrophic scars and post‐inflammatory hyperpigmentation, similar to the case presented here. However, the current case demonstrated more severe atrophic scarring and persistent hyperpigmentation, with only modest improvement achieved despite laser intervention. This case highlights the risks associated with the use of unapproved products, emphasizing the importance of regulatory compliance and adherence to manufacturer instructions. It also underscores the need for further research into the safety and efficacy of exosome‐based therapies before their widespread adoption in dermatology and aesthetic medicine.

## Author Contributions

Salma AlBargawi: conceptualization, methodology, investigation, data analysis, writing – original draft, and writing – review and editing.

## Ethics Statement

Written informed consent was obtained from the patient for this case presentation and any accompanying images.

## Consent

Written informed consent was obtained from the patient of this case presentation and any accompanying images.

## Conflicts of Interest

The author declares no conflicts of interest.

## Data Availability

The data that support the findings of this study are available from the corresponding author upon reasonable request.
